This article has been retracted.

# Effects of High Flux Hemodialysis Combined with L-Carnitine on Microinflammation and Arteriovenous Fistula in Maintenance Hemodialysis Patients

**DOI:** 10.1155/2022/6964127

**Published:** 2022-07-05

**Authors:** Yunhong Zhou

**Affiliations:** Department of Hemodialysis, East District, Lujiang County People's Hospital, Hefei, China

## Abstract

**Objective:**

To explore the effects of high-flux hemodialysis combined with L-carnitine on microinflammation and arteriovenous fistulas in maintenance hemodialysis patients.

**Methods:**

A total of 65 patients admitted to our hospital from May 2017 to May 2019 were selected and divided into a control group of 30 cases and an experimental group of 35 cases according to the selected treatment plan. Combined with L-carnitine, the cardiac function of the two groups of patients before and after the treatment was evaluated, the microinflammatory indexes of the two groups were compared, and the clinical efficacy of the combined treatment on MHD patients was analyzed.

**Results:**

The two groups were not significantly different in general information such as age, gender, course of disease, and past medical history (*P* > 0.05). The experimental group generated a notably higher total effective rate of treatment in relation to the control group (*P* < 0.05). After treatment, lower heart function levels of LVST and LEVDD were observed in the experimental group as compared to the control group, but LVEF was higher than that in the control group (*P* < 0.05). The GQOLI-74 score of the experimental group was better than that of the control group (*P* < 0.05). The incidence of venous fistula complications in the experimental group was significantly lower than that in the control group (*P* < 0.05). The microinflammatory index hs-CRP in the experimental group was lower (*P* < 0.05) and the microinflammatory index TNF-*α* was significantly lower (*P* < 0.05). The HAD score after treatment of the experimental group was better than that of the control group (*P* < 0.05).

**Conclusion:**

High-flux hemodialysis combined with L-carnitine therapy has achieved satisfactory results in patients with MHD in terms of alleviating the level of inflammatory factors, improving heart function, enhancing patients' living standards, reducing complications of intravenous fistula, and boosting the prognosis. It is worthy of promotion.

## 1. Introduction

Maintenance hemodialysis (MHD), a commonly used renal replacement therapy, can be guaranteed by ensuring the continuous operation of vascular access [1, 2]. The purpose of hemodialysis is to replace some of the functions lost in renal failure, maintain electrolyte balance, and remove metabolic waste [3]. Studies have pointed out that long-term MHD treatment can cause microinflammation in the patient's body of microorganisms, immune complexes, and various chemical drugs. It can also affect intravenous fistulas, cause complications, and seriously affect the prognosis outcome [4]. Numerous documents have confirmed that long-term dialysis treatment can easily lead to negative emotions in patients, reduce dialysis tolerance, and also develop various diseases such as microinflammation, which threaten the life safety of patients. With the improvement of the medical level, the clinic has put forward higher requirements for MHD, not only to maintain the life of the patient and prolong the life span, but also to enhance the quality of life of the patient and improve the psychological state of the patient [5, 6].

An intravenous fistula is a frequently used vascular access for MHD patients. However, in practical applications, venous fistulas are prone to thrombosis and obstruction, leading to adverse symptoms such as insufficient dialysis and microinflammation, which in turn affect cardiac function. To reduce microinflammation and the impact on intravenous fistulas, high-flux hemodialysis combined with L-carnitine was used for joint intervention [7, 8]. High-flux dialysis is a new blood purification technique that uses high-flux hemodialyzers to replace ordinary hemodialyzers for hemodialysis treatment. It has the advantage of removing more medium molecular weight toxins [9]. L-carnitine is a natural substance in the body necessary for energy metabolism in mammals. Its main function is to promote lipid metabolism and relieve myocardial dysfunction. The combination of the two can improve the effect of MHD [10, 11]. This study intends to investigate the effects of high-flux hemodialysis combined with L-carnitine on microinflammation and arteriovenous fistulae in patients with MHD, using 65 patients admitted to our hospital from May 2017 to May 2019 as observation subjects.

## 2. Materials and Methods

### 2.1. Ethical Statement

The study was approved by the Ethics Committee of Lujiang County People's Hospital (no. 1077713), and the patients and their families were informed of the purpose and process of the experimental study and signed the informed consent.

### 2.2. General Information

Altogether, 65 patients treated in our hospital from May 2017 to May 2019 were recruited as research subjects. After screening, all patients met the research conditions. According to the treatment plan, they were divided into an experimental group and a control group. Among them, there were 30 patients in the control group and 35 in the experimental group.

### 2.3. Inclusion Criteria

① All met the diagnostic criteria of this disease in the *Guide to Nephropathy* [12], with clinical glomerulosclerosis, pyknosis, blood creatinine increase greater than 707 *μ*mol/L, endogenous creatinine clearance rate decreased by 15 mL/min. ② Complete data. ③ No allergic symptoms to the drugs used. ④ Patients and their family members were aware of this study, and they signed an informed consent form under the premise of knowing the purpose and process, and the study has been approved by the hospital ethics committee.

### 2.4. Exclusion Criteria

① With other dysfunctional diseases. ② Cognitive and social disorders and refused to cooperate with the experiment. ③ Participated in a similar study in other hospitals. ④ Intolerant to treatment.

### 2.5. Treatment Methods

Both groups were given recombinant human erythropoietin, folic acid, and other drugs on the basis of blood pressure control to improve nutritional status and maintain water and electrolyte balance [13].

The control group carried out high-flux hemodialysis treatment: the high-flux polysulfide membrane hollow fiber selects the German Fresenius FX80 flux dialyzer; specification: Fx80; model: Fx80; membrane area: 1.8; wall thickness: 45; inner diameter: 185 [14].

The experimental group received high-flux hemodialysis combined with L-carnitine treatment: the high-flux hemodialysis treatment was the same as the control group; L-carnitine (Chinese Medicine Standard: H20000543, Manufacturer: Changzhou Lanling Pharmaceutical Co., Ltd., Specification: 5 ml : 1 g) was intravenously administered; at the end of each hemodialysis, 1 g of this product was diluted with 15 ml of normal saline, and slowly injected for 2 to 3 min. The treatment was given 3 times a week for 3 months [15, 16].

### 2.6. Efficacy Criteria

1. Clinical efficacy: Cured is defined if the patient's NIHSS score decreased by ≥90% after treatment; markedly effective is considered if the NIHSS score decreased by 45%–90% after treatment; improved is deemed if the NIHSS score decreased by 8%–44% after treatment; ineffective is regarded if the NIHSS reduced by less than 8% after treatment. The total effective rate = cured rate + markedly effective + improved rate.
2. Cardiac function indexes: End-diastolic ventricular septal thickness (LVST), left ventricular ejection fraction (LVEF), and left ventricular end-diastolic diameter (LEVDD) before and after the treatment were compared between the two groups.
3. Quality of life: The Generic Quality of Life Inventory-74 (GQOLI-74) [17] was used to assess the quality of life of the two groups of patients after treatment. The scale was scored from the dimensions of mental function, physical function, social function, and material life state, and the total score is 100 points. The higher the score, the better the quality of life of the patients.
4. Complications of Intravenous Fistula: Complications including muscle spasm, fistula infection, and vascular sclerosis were compared.
5. Microinflammatory indicators: Serum high-sensitivity C-reactive protein (hs-CRP), tumor necrosis factor-*α* (TNF-*α*), and interleukin-6 (IL-6) levels) before and after the treatment in the two groups were compared. 3 ml of blood sample was collected from the patient in the fasting state in the early morning of the next day, and the levels of hs-CRP, TNF-*α*, and IL-6 were measured with an automatic immunoluminescence analyzer. The kit was purchased from Shanghai Enzyme Link Biotechnology Co., Ltd., and the operation was performed in accordance with the kit instructions.
6. HAD mood measurement scale [18] was used to assess the emotional state of patients before and after the treatment. The total score on the scale is 42 points. The higher the score, the more severe the anxiety and depression of the patient.

### 2.7. Statistical Methods

Statistical analysis was performed with the SPSS 23.0 version software. Counting data were expressed as percentage [*n* (%)] and examined by the *X*2 test; measurement data were expressed as mean ± standard deviation ($\bar{x}\pm s$), and analyzed by the *t*-test. Values of *P* < 0.05 indicates that the difference is statistically significant.

## 3. Results

### 3.1. Comparison of General Information between the Two Groups

The two groups were not significantly different in general information such as age, gender, course of disease, and past medical history (*P* > 0.05). See Table 1.

### 3.2. Comparison of Clinical Efficacy between the Two Groups

The total efficiency of the control group was 67%, and the total efficiency of the experimental group was 97%. The experimental group generated a notably higher total effective rate of treatment in relation to the control group (*P* < 0.05), see Table 2.

### 3.3. Comparison of the Cardiac Function Indexes before and after Treatment between the Two Groups

After treatment, lower heart function levels of LVST (after treatment, the experimental group was 52.13 ± 6.67%, and the control group was 43.21 ± 5.21%) and LEVDD (the experimental group was 51.25 ± 5.24 mm after treatment, and the control group was 59.62 ± 5.72 mm) were observed in the experimental group as compared to the control group, but LVEF (the experimental group was 8.85 ± 1.06 mm after treatment, and the control group was 11.24 ± 1.13 mm) was higher than that in the control group (*P* < 0.05), as shown in Table 3.

### 3.4. Comparison of the GQOLI-74 Scores of the Two Groups

The psychological function score of the experimental group was 82.44 ± 5.72, and that of the control group was 75.12 ± 5.18. The physiological function score of the experimental group was 86.28 ± 5.78, and that of the control group was 64.22 ± 5.45. The social function score of the experimental group was 87.25 ± 6.53, and that of the control group was 66.88 ± 4.25. The material life status score of the experimental group was 88.63 ± 6.78, and that of the control group was 65.25 ± 5.72. The scores of all indicators of GQOLI-74 score in the experimental group were better than those in the control group (*P* < 0.05), as shown in Table 4.

### 3.5. Comparison of Complications of Intravenous Fistula between the Two Groups

The experimental group experienced an evidently lower complication rate of intravenous fistula than the control group (*P* < 0.05), as shown in Figure 1.

### 3.6. Comparison of hs-CRP Levels before and after Treatment between the Two Groups

Figure 2 shows that the experimental group experienced lower microinflammatory index hs-CRP in comparison with the control group (*P* < 0.05).

### 3.7. Comparison of the TNF-*α* Levels of the Two Groups before and after Treatment

A remarkably lower level of microinflammation index TNF-*α* in the experimental group was witnessed than that in the control group (*P* < 0.05), as presented in Figure 3.

### 3.8. Comparison of the Levels of IL-6 before and after the Treatment in the Two Groups

The level of IL-6, an indicator of microinflammation in the experimental group, was lower than that in the control group (*P* < 0.05), see Figure 4.

### 3.9. Comparison of the HAD Scores of the Two Groups before and after Treatment

Figure 5 displays that the HAD score after treatment of the experimental group was better than that of the control group (*P* < 0.05).

## 4. Discussion

MHD is a common technique for the clinical treatment of renal failure, which uses hemodialysis or peritoneal dialysis to save the lives of patients and extend their life cycle. With the increasing incidence of end-stage renal disease, MHD has become more and more widely used. On the one hand, microinflammation can affect the cardiovascular function of patients, which can easily aggravate the degree of renal failure, lead to malnutrition, and greatly reduce the quality of life [19, 20]. The microinflammatory state is a neutral link in the occurrence of cardiovascular and cerebrovascular events, malnutrition, and the promotion of red pigment resistance in MHD patients. On the other hand, it is also a key factor affecting residual renal function and dialysis adequacy [21]. Microinflammation is the result of the continuous activation of the macrophage system. TNF-*α* is a tumor necrosis factor that can kill some tumor cells or cell lines both in vivo and in vitro. It is mainly caused by activated monocytes, macrophages, and other cells. It has a certain relationship with the heart, liver, kidney, and heart failure due to the extremely complex biological activity. IL-6 is a lymphokine produced by activated T cells and fibroblasts. It is a proinflammatory cell mediator and plays an important role in the inflammatory response. hs-CRP is a nonspecific marker in the acute phase of systemic inflammatory response, an important indicator for the diagnosis of microinflammation, and has a certain effect on the prognosis of MHD [22, 23].

In modern clinical research, in-depth research on the mechanism of maintenance hemodialysis has been increased, and certain progress has been obtained. It has been found that the inflammation affecting MHD patients is due to incomplete clearance of inflammatory factors combined with inadequate hemodialysis, which leads to microinflammation and thus affects intravenous fistulas. High-flux hemodialysis is a new type of high-permeability filter that can eliminate small molecules, excess water in the body, and metabolic waste through diffusion, ultrafiltration, adsorption, etc., effectively reducing microinflammation and protecting heart function and reducing cardiovascular morbidity. However, the use of a single high-flux hemodialysis cannot achieve the expected results. L-carnitine is a natural substance in the body necessary for energy metabolism in mammals. Its main function is to promote lipid metabolism and its oxidative decomposition, providing energy for cells, improving oxidative stress, and, moreover, inhibiting inflammatory factors [24].

The results of this study confirmed that the total effective rate of treatment in the experimental group was higher than that in the control group, indicating that the combined application of the two can improve the treatment effect and improve the prognosis. After treatment, the heart function levels of LVST and LEVDD in the experimental group were lower than those in the control group, but the LVEF was higher than that in the control group, suggesting that the combination of the two improved the heart function and helped reduce the incidence of cardiovascular disease. The GQOLI-74 score of the experimental group was better than that of the control group, confirming that the combination of high-flux hemodialysis combined with L-carnitine improved the quality of life of the patients, which is of great significance for accelerating the recovery of the patient's body. Additionally, the complication rate of intravenous fistula in the experimental group was observed to be lower than that in the control group, which played an important role in the value of intravenous fistula. Moreover, after treatment, the levels of hs-CRP, TNF-*α,* and IL-6 in the experimental group were lower than those in the control group, which was consistent with the results of Nicos et al. [25] (2019), who pointed out that lower TNF-*α* (*P* < 0.01) and IL-6 (*P*=0.01) were witnessed in the observation group, indicating that the combined application of the two can reduce the level of inflammatory factors and mitigate the state of micro-inflammation. Remarkably, the HAD score of the experimental group after treatment was superior to that of the control group, implying that the combined application can relieve negative emotions, promote prognosis, and is conducive to recovery.

L-carnitine is a special amino acid that is important in the beta-oxidation of fatty acids. Carnitine deficiency in hemodialysis patients is due to insufficient carnitine synthesis, especially when it is lost during dialysis. Human body functions gradually degrade with age, so elderly patients are more susceptible to L-CN deficiency, which exacerbates complications such as dialysis hypotension, myocardial damage, and renal anemia. Therefore, improving the quality of dialysis in elderly patients and reducing dialysis complications is an urgent task in clinical research. Studies have shown that the application of L-CN has greatly improved living standards and dialysis quality, and follow-up experiments can be considered to study the feasibility of preventing complications by preadministering L-CN [26].

It is worth mentioning that more and more people are now trusting traditional Chinese medicine (TCM) as it is increasingly showing its unique advantages in the treatment system. Chinese medicine also plays a unique role in the treatment of chronic kidney disease. For example, there are different treatment options for different stages of development of chronic kidney disease, and TCM is effective in stopping the progression of kidney disease from getting worse. Chinese medicine plays a pivotal role in the nondialysis treatment of chronic renal failure following abnormal kidney function. For patients on hemodialysis, based on regular dialysis, correction of anemia with western drugs, lowering of blood pressure, and calcium supplementation, Chinese medicine is given appropriately according to the patient's different clinical manifestations and has a very good effect on prolonging the patient's life and relieving the patient's suffering.

The combination of high throughput hemodialysis and L-carnitine in the treatment of MHD patients was found to have satisfactory results in reducing inflammatory factors, improving cardiac function, improving patients' standard of living, reducing the complications of intravenous fistula, and improving prognosis. Therefore it is worthy of clinical promotion. However, since the number of samples is too small, and recovery is a long process, there are certain contingencies, which should be improved and further analyzed in follow-up experiments.

## Figures and Tables

**Figure 1:** Comparison of complications of intravenous fistula between the two groups. Black represents muscle spasm; dark gray represents internal fistula infection; light gray represents vascular sclerosis; and white represents no complications. (a) The complications in the experimental group included 1 case of muscle spasm (2.86%), 1 case of internal fistula infection (2.86%), 1 case of vascular sclerosis (2.86%), and 32 cases (91.42%) without complications, and the total number of complications patients was 3 (8.58%). (b) The complications in the control group included 2 cases of muscle spasm (6.67%), 5 cases of internal fistula infection (16.66%), 2 cases of vascular sclerosis (6.67%), and 21 cases (70%) without complications, and the total number of complications patients was 9 (30%). There was a significant difference in the incidence of adverse reactions between the two groups (*x*^2^ = 4.928, *P* < 0.05).

**Figure 2:** Comparison of hs-CRP levels before and after the treatment between the two groups ($\bar{\chi }\pm S$). The abscissa indicates before and after the treatment, and the ordinate indicates the level of hs-CRP, ng/L. The hs-CRP levels of the experimental group before and after the treatment were (8.95 ± 0.86) ng/L and (3.26 ± 0.34) ng/L, respectively; the hs-CRP levels of the control group before and after treatment were (8.86 ± 0.97) ng/L and (5.75 ± 0.63) ng/L, respectively; ^*∗*^hs-CRP levels of the experimental group were different before and after the treatment (*t* = 34.002, *P* < 0.001); ^*∗∗*^hs-CRP levels of the control group before and after the treatment are different (*t* = 15.043, *P* < 0.001); ^*∗∗∗*^difference in hs-CRP levels between the two groups after treatment (*t* = 20.215, *P* < 0.001).

**Figure 3:** Comparison of TNF-*α* levels before and after the treatment in the two groups ($\bar{\chi }\pm S$). The abscissa indicates before and after the treatment, and the ordinate indicates the level of TNF-*α*, pmol/L. The levels of TNF-*α* in the experimental group before and after the treatment were (28.35 ± 8.24) pmol/L and (18.26 ± 6.34) pmol/L; the TNF-*α* levels of the control group before and after the treatment were (28.42 ± 8.06) pmol/L and (24.75 ± 6.43) pmol/L; ^*∗*^difference in the level of TNF-*α* in the experimental group before and after the treatment (*t* = 5.461, *P* < 0.001); ^*∗∗*^there is a difference in the level of TNF-*α* in the control group before and after the treatment (*t* = 2.006, *P* < 0.001); ^*∗∗∗*^difference in the levels of the two groups after treatment (*t* = 4.087, *P* < 0.001).

**Figure 4:** Comparison of IL-6 levels before and after the treatment between the two groups (±*S*). The abscissa indicates before and after the treatment, and the ordinate indicates the level of IL-6, ng/L. The IL-6 levels of the experimental group before and after the treatment were (18.34 ± 3.24) ng/L and (10.26 ± 2.12) ng/L; the IL-6 levels of the control group before and after the treatment were (18.32 ± 3.28) ng/L and (14.54 ± 2.36) ng/L; ^*∗*^indicates that there is a difference in IL-6 levels in the experimental group before and after the treatment (*t* = 11.677, *P* < 0.001); ^*∗∗*^there is a difference in the IL-6 level of the control group before and after the treatment (*t* = 5.251, *P* < 0.001); ^*∗∗∗*^there is a difference in IL-6 levels between the two groups after treatment (*t* = 7.701, *P* < 0.001).

**Figure 5:** Comparison of the HAD scores of the two groups before and after the treatment ($\bar{x}\pm s$, point). The abscissa represents before and after the treatment, and the ordinate represents the HAD score, points; the HAD scores of the patients in the experimental group before and after intervention were (37.51 ± 3.25) points and (6.46 ± 1.23) points, respectively. The HAD scores of the control group before and after intervention were (37.38 ± 3.12) points and (15.29 ± 2.63) points, respectively; ^*∗*^there is a significant difference in the HAD scores of the experimental group before and after intervention (*t* = 49.342, *P* < 0.001); ^*∗∗*^that there is a significant difference in the HAD scores of the control group before and after intervention (*t* = 30.565, *P* < 0.001); ^*∗∗∗*^that there is a significant difference in the HAD scores of the two groups of patients after intervention (*t* = 17.744, *P* < 0.001).

**Table 1:** Comparison of general information of the two groups.

	Experimental group (*n* = 35)	Control group (*n* = 30)	*t*/*χ*^2^	*P*
Age (year)	51.24 ± 6.43	52.03 ± 6.87	0.478	0.634

Gender (male/female)	20/15	17/13	0.002	0.969

Course of disease (year)	2.12 ± 1.24	2.36 ± 1.18	0.795	0.429

Dialysis time (month)	10.36 ± 5.42	10.78 ± 5.14	0.319	0.751

Past medical history			0.006	0.939
Diabetic nephropathy (%)	16 (45.71)	14 (46.67)		
Hypertensive nephropathy (%)	19 (54.29)	16 (53.33)		

Place of residence			0.054	0.816
Township (%)	20 (57.14)	18 (60)		
Rural area (%)	15 (42.86)	12 (40)		

Drinking			0.000	1.000
Yes (%)	14 (40)	12 (40)		
No (%)	21 (60)	18 (60)		

Smoking			0.029	0.864
Yes (%)	10 (28.57)	8 (26.67)		
No (%)	25 (71.43)	22 (73.33)		

**Table 2:** Comparison of the clinical efficacy of the two groups [*n* (%)].

Groups	*n*	Cured	Markedly effective	Improved	Ineffective	Total effectiveness
Experimental group	35	10	14	10	1	97% (34/35)
Control group	30	2	6	12	10	67% (20/30)
*χ* ^2^						10.672
*P*						0.001

**Table 3:** Comparison of the cardiac function indexes of the two groups before and after the treatment ($\bar{\chi }\pm S$).

	Time	Experimental group (*n* = 35)	Control group (*n* = 30)	*t*	*P*
LVST (mm)	Before treatment after treatment	13.24 ± 1.26 8.85 ± 1.06	12.98 ± 1.42 11.24 ± 1.13	0.782 8.790	0.437 <0.001

LVEF (%)	Before treatment after treatment	36.56 ± 5.31 52.13 ± 6.67	36.48 ± 5.52 43.21 ± 5.21	0.059 5.934	0.953 <0.001

LEVDD (mm)	Before treatment after treatment	62.24 ± 5.37 51.25 ± 5.24	61.86 ± 5.68 59.62 ± 5.72	0.277 6.154	0.783 <0.001

**Table 4:** Comparison of the GQOLI-74 scores of the two groups ($\bar{x}\pm s$ point).

Group	*n*	Mental function	Physical function	Social function	State of material life
Experimental group	35	82.44 ± 5.72	86.28 ± 5.78	87.25 ± 6.53	88.63 ± 6.78
Control group	30	75.12 ± 5.18	64.22 ± 5.45	66.88 ± 4.25	65.25 ± 5.72
*T*		5.371	15.747	14.627	14.882
*P*		<0.001	<0.001	<0.001	<0.001

## Data Availability

The data used to support the findings of this study are available from the corresponding author upon request.
